# Predictors of Quality of Life Among People Living With Multimorbidity in Karachi, Pakistan: A Cross-Sectional Study

This article has been retracted.

**DOI:** 10.7759/cureus.18803

**Published:** 2021-10-15

**Authors:** Malik Hatim Hussain, Daniyal A Jilanee, Safa Aziz, Sheharyar Tariq, Arti Devi, Camilo A Avendaño-Capriles, Sohaib Tousif, Rahil Barkat

**Affiliations:** 1 Orthopaedics and Trauma, East Lancashire NHS Hospitals, Blackburn, GBR; 2 Medicine, Liaquat National Hospital and Medical College, Karachi, PAK; 3 Medicine, Ziauddin University, Karachi, PAK; 4 Medicine, Lahore Medical and Dental College, Lahore, PAK; 5 Medicine, Harvard Medical School, Boston, USA; 6 Medicine, Universidad del Norte, Barranquilla, COL; 7 Epidemiology, Indus Hospital Research Center, The Indus Hospital, Karachi, PAK

**Keywords:** quality of life, chronic disease, karachi, multimorbidity, predictors

## Abstract

Introduction

Multimorbidity is defined as the coexistence of more than one chronic condition in one individual. It is related to enhanced rates of disability and mortality, enhanced disease burden, decreased function levels, and it can affect the wellbeing and daily activities of people, including loss of autonomy and independence. The aim of the current study is to determine the predictors of quality of life among patients with multimorbidity in Karachi, Pakistan.

Methodology

It was a cross-sectional study conducted in 12 health care facilities of six districts in Karachi, Pakistan. Two health care facilities were selected from each district using a convenient sampling technique. The total sample size of this study was 690, equally distributed among 12 health care facilities.

Results

The majority of participants (33.47%) belonged to the age group of 40 to 49 years, while 29.85% of participants had an age between 30 to 39 years. More than half of the participants were females (50.87%). Overall, the multivariate analysis showed being male, married, younger, high educational status and employed were positively associated with quality of life. While having lower family income is negatively associated with quality of life.

Conclusion

The findings of this study had important implications for identifying distinct multimorbidity individuals who were at risk of a lower quality of life, and they emphasized the need for disease detection and treatment at an early stage. The study can also give important evidence for decision-makers when it comes to allocating health resources more efficiently, and health administrative departments can improve chronic disease management.

## Introduction

Multimorbidity is defined as the coexistence of more than one chronic condition in one individual [1]. It is related to enhanced rates of disability and mortality, enhanced disease burden, decreased function levels, and it can affect the wellbeing and daily activities of people, including loss of autonomy and independence [2]. All these factors create negative impacts on the quality of life of people who suffer from multimorbidity. Chronic diseases are viewed as chiefly affecting old age people. In fact, those under the age of 60 account for a fifth of all chronic disease deaths. Furthermore, multimorbidity is common among adults (20 to 64 years old) all over the world [3]. The impact created by multimorbidity on quality of life of people is severe than we imagined.

Different studies in developed countries have presented that magnitude of multimorbidity is increasing with the prevalence of 25% to 60% in community and health care settings [4,5]. On the other hand, the situation related to multimorbidity in lower and middle-income countries is unclear. Amongst low and middle-income countries, Pakistan, one of the largest demographics in the world, is experiencing an upward movement in life expectancy, non-communicable diseases burden is increasing along with communicable diseases, and they are acting as the contributors to mortality and morbidity [6]. Quality of life is a vital indicator to assess the outcomes of treatment programs. Different studies have indicated that the quality of life of patients with multimorbidity is poor as compared to normal people [7].

The study conducted by Bao et al. found that patients with chronic diseases were related to worse health-related quality of life in a sample of Chinese middle-aged and elderly adults [8]. The study found that different combinations and types of chronic diseases reduced health-related quality of life in varying degrees and that this decline continued even after controlling for confounding factors. Although hypertension has the highest prevalence, it has the least influence on Health-related Quality of life (HRQoL). The reduction in HRQoL is highest when chronic pain and bone disease are combined. Furthermore, certain chronic disorders, particularly those involving hypertension or dyslipidemia, frequently occurred in pairs. In addition, different factors can affect the quality of life of patients with multimorbidity, including age, gender, educational status, and monthly income [8,9,10].

Multimorbidity can create a negative impact on the quality of life and considering the significance of quality of life in patients outcomes along with the lack of literature related to the predictors of quality of life in the Pakistani population, we conducted a cross-sectional study among the adults in Karachi, Pakistan. The aim of the current study is to determine the predictors of quality of life among patients with multimorbidity in Karachi, Pakistan.

## Materials and methods

This was a cross-sectional study conducted in 12 health care facilities of six districts in Karachi, Pakistan. Two health care facilities were selected from each district using a non-probability convenient sampling technique. We included private primary health care facilities as a large number of people in Karachi consult private practitioners for health care. Ethical approval for this study was taken from the Institutional Review Board of Liaquat National Hospital with an IRB number of 2021_03_12. Informed consent was taken from all participants prior to their enrollment. 

Sample size and study participants

The sample size was calculated based on the study conducted in India by Pati et al. [9]. Considering that 28.6% of patients attending primary health care settings have multimorbidity, the sample was calculated to be 690 considering the design effect of 2.0 and the non-response rate of 10%. It was decided to divide this sample size equally among all selected health care facilities to cover a diverse population i.e. 58 participants. Participants were enrolled in the study using non-probability consecutive sampling techniques from each health care facility until the desired sample was achieved. Selected patients were interviewed after the consultation with a doctor to avoid any disturbance and delays to the hospital management system.

Inclusion and exclusion criteria

Participants were eligible if they had two or more chronic conditions, having age 18 years or more, and were ready to be a part of the study. Patients too ill to the participant and those with the insufficient cognitive ability to give appropriate responses to the questions, and those with mental disabilities and physical disabilities and were unwilling to participate in the study were excluded.

Data collection instrument

The data was collected using the pre-designed survey questionnaire (see Appendices). The multimorbidity was determined by self-report as a yes or no response to the question stem, "Has a doctor ever diagnosed that you had…." [11] In the study, 19 diseases were investigated that included phthisis, depression, anxiety, dementia, multiple sclerosis, cancer, chronic kidney disease, chronic obstructive pulmonary disease, gallbladder and spleen disease, stroke, peripheral vascular disease, coronary disease, gout, gastroenteritis, dyslipidemia, diabetes mellitus, bones diseases, chronic pain, and hypertension. Open options were for additional conditions, if any, to be added by the participant. Trained data collectors verified the chronic illness of the study participants through the medications and the diagnosis results in order to make sure the comprehensiveness and authenticity of the interview.

The sociodemographic part of the survey questionnaire assessed information on age, gender, educational status, marital status, ethnicity and family monthly income in PKR (Pakistani Rupees). The abbreviated World Health Organization Quality of Life (WHOQOL-BREF) questionnaire was used to assess the quality of life among participants. The WHOQOL-BREF questionnaire is available in different languages, and in the current study, the Urdu version was used for assessing the quality of life. It is a valid questionnaire, which is composed of 26 questions, of which 24 were grouped into four domains, including physical, psychological, social relations, and environment, while the remaining two questions have assessed satisfaction and self-perceived quality of life with health [12]. In the current study, we only assessed four domains of quality of life, therefore 24 questions assessing physical, psychological, social relations, and environment were used in the study. Each of the above domains is represented by several questions and facets and are created for a Likert scale, with capacity (nothing - completely), intensity (nothing - extremely), frequency (never - always), and assessment scales (very dissatisfied - very satisfied; very bad - very good), all of them consisting of five levels (1 to 5) [12]. Scores obtained were converted into a transformed score that directly converted the raw scores into the transformed domains. Five-level scores are more reliable due to their ability to measure intermediary and extremes accessibility scores [13].

Data analysis

Data were analyzed by using STATA Windows version 16.0 (StataCorp, College Station, USA). Mean and standard deviation were calculated for continuous variables, while categorical variables were presented as frequency and percentages. ANOVA and Independent t-test was performed to compare the different scores of domains of quality of life among different participants characteristics. All the factors associated were further examined by multivariable linear regression using the stepwise forward approach with a cut-off point for p-value at 0.05. For statistical analysis in the four domains, transformed scores were used.

## Results

The characteristics of participants are shown in Table 1. Most of the participants (33.47%) in the study belonged to the age group of 40 to 49 years, while 29.85% of participants had an age between 30 to 39 years, 50.87% were females, 85.79% were married, 53.19% were speaking Urdu as a mother tongue, 37.68% had at least bachelors degree, and 64.35% were employed. Hypertension (35%), diabetes (32%), and arthritis (20%) were the most common comorbidities among the study participants.

**Table 1:** Characteristics of Participants (N=690) PKR: Pakistani Rupees

Variable	n(%)
Age	
30-39 years	206 (29.85)
40-49 years	231 (33.47)
50-59 years	74 (10.72)
60-69 years	119 (17.24)
>=70 years	60 (8.69)
Gender	
Male	339 (49.13)
Female	351 (50.87)
Marital Status	
Never married	44 (6.38)
Currently married	592 (85.79)
Seprated/Divorced	54 (7.83)
Ethnicity	
Sindhi	103 (14.93)
Punjabi	65 (9.42)
Balochi	25 (3.62)
Pashtu	43 (6.23)
Urdu	372 (53.91)
Others	82 (11.88)
Monthly Income	
>10000 PKR	34 (4.92)
10000-20000 PKR	164 (23.76)
20000-30000 PKR	179 (25.94)
30000-40000 PKR	226 (32.75)
>40000 PKR	87 (12.61)
Employment Status	
Employed	444 (64.35)
Unemployed	246 (35.65)
Educational Status	
Illiterate	59 (8.55)
Under secondary school	220 (31.88)
Under Intermediate	151 (21.88)
at least bachelors	260 (37.68)

Table 2 presents the WHOQOL-BREF mean score of four domains. The highest mean score of satisfaction was found in the social relationship (Domain 3), with a mean score of 63.74 and an SD of 19.94. On the other hand, the lowest mean score was found in the environment domain, with a mean of 58.13 (±13.97).

**Table 2:** Domains of Quality of life QOL: quality of life; DOM: domain

QOL Domains	Mean (SD)
Physical (DOM1)	61.43 (15.28)
Psychological (DOM2)	62.19 (15.11)
Social relationships (DOM3)	63.74 (19.94)
Environment (DOM4)	58.13 (13.97)

The mean score of each domain across characteristics of participants is presented in Table 3. The means of all four domains were significantly different across gender, monthly family income, employment status, and marital status. In addition, mean scores of domain physical, psychological and social relationships are different across age groups and educational status, while ethnicity was significantly different in environmental health.

**Table 3:** Mean score of each domain across characteristics of participants * Significant at ≤0.05 DOM: domain; PKR: Pakistani Rupees

Variable	Physical (DOM1) Mean (SD)	p-value	Psychological (DOM2) Mean (SD)	p-value	Social relationships (DOM3) Mean (SD)	p-value	Environment (DOM4) Mean (SD)	p-value
Age								
30-39 years	62.53 (15.32)	0.001*	64.07 (14.49)	0.005*	66.99 (17.72)	0.001*	58.98 (14.07)	0.511
40-49 years	63.32 (14.45)		62.84 (14.65)		66.23 (18.64)		57.91 (13.71)	
50-59 years	61.96 (14.71)		63.56 (13.53)		64.07 (22.32)		58.91 (12.63)	
60-69 years	58.37 (16.63)		58.72 (16.19)		57.98 (21.51)		57.93 (15.47)	
>=70 years	55.45 (14.25)		58.18 (17.23)		53.50 (20.71)		55.37 (13.1)	
Gender								
Male	65.05 (14.22)	0.001*	64.89 (14.19)	0.001*	66.29 (17.24)	0.001*	59.16 (12.64)	0.029*
Female	57.96 (15.48)		59.60 (15.52)		61.30 (21.97)		57.14 (15.09)	
Marital Status								
Never married	65.15 (4.80)	0.006*	66.36 (14.08)	0.005*	60.77 (20.51)	0.001*	62.42 (10.53)	0.044*
Currently married	61.83 (15.11)		62.40 (15.07)		65.42 (18.43)		58.10 (14.14)	
Seprated/Divorced	54.23 (15.65)		56.63 (15.04)		47.53 (27.11)		55.20 (13.73)	
Ethinicity								
Sindhi	61.19 (15.13)	0.426	62.01 (13.39)	0.181	62.45 (18.73)	0.215	53.58 (12.66)	0.001*
Punjabi	60.21 (15.35)		60.06 (16.89)		62.82 (20.99)		56.92 (16.10)	
Balochi	66.39 (13.43)		66.47 (13.57)		71.96 (14.44)		57.38 (13.55)	
Pashtu	59.96 (15.55)		58.52 (14.31)		62.98 (20.91)		52.90 (11.45)	
Urdu	62.00 (15.27		63.08 (15.15)		64.56 (19.78)		60.29 (13.49)	
Others	59.53 (15.77)		60.82 (15.96)		60.56 (21.71)		57.96 (15.30)	
Monthly Income								
>10000 PKR	52.30 (13.12)	0.005*	59.13 (14.41)	0.022*	55.91 (24.36)	0.021*	52.82 (16.08)	0.001*
10000-20000 PKR	59.18 (15.12)		58.68 (16.48)		61.58 (20.99)		54.87 (14.49)	
20000-30000 PKR	62.60 (15.28)		62.24 (14.77)		63.26 (19.80)		56.61 (13.84)	
30000-40000 PKR	63.52 (15.34)		64.63 (13.31)		66.62 (18.58)		61.14 (12.71)	
>40000 PKR	61.04 (14.71)		63.40 (16.58)		64.08 (19.03)		61.45 (13.38)	
Employment Status								
Employed	64.81 (13.91)	0.001*	65.58 (13.20)	0.001*	66.59 (19.08)	0.001*	59.79 (12.97)	0.001*
Unemployed	55.24 (15.76)		55.98 (16.38)		58.53 (20.46)		55.10 (15.21)	
Educational Status								
Illiterate	53.66 (13.21)	0.001*	56.29 (13.44)	0.001*	55.48 (12.78)	0.002*	59.82 (17.32)	0.149
Under secondary school	58.15 (13.62)		59.78 (13.56)		61.26 (13.55)		60.61 (17.68)	
Under Intermediate	58.59 (14.25)		60.02 (14.62)		63.27 (17.68)		60.22 (18.63)	
at least bachelors	66.37 (14.33)		66.18 (15.12)		66.18 (16.58)		61.56 (13.58)	

The results of multivariable linear regression are shown in Table 4. Table 4 presents the coefficient and 95% CI of only those variables that were significantly associated with each domain of quality of life. The reference group of each independent categorical variable was compared with all the dummy variables of that specific categorical variable to assess the difference of scores between groups. After adjusting all the other variables in the model, employment status is the only factor statistically significantly associated with all four domains of quality of life. Age and gender were associated with physical health, psychological health, and social relationships. Educational status was associated with psychological and physical health domains. The monthly family income was significantly associated with physical health and environmental health. Similarly, marital status was only associated with social relationships. Overall, the multivariate analysis showed being male, married, younger, and employed were positively associated with quality of life. While belonging to lower socioeconomic status is negatively associated with quality of life.

**Table 4:** Multiple linear regression of factors significantly associated with domains of quality of life DOM: domain; PKR: Pakistani Rupees; B: beta coefficient

Variable	Physical (DOM1)		Psychological (DOM2)		Social relationships (DOM3)		Environment (DOM4)	
	B(95% CI)	p-value	B(95% CI)	p-value	B(95% CI)	p-value	B(95% CI)	p-value
Age								
30-39 years	Reference Group							
40-49 years	-0.69 (-3.38, 1.99)	0.611	-2.97 (-5.65, -0.29)	0.030	-3.04 (-6.61, 0.52)	0.094		
50-59 years	-1.98 (-5.74, 1.77)	0.301	-2.10 (-5.87, 1.67)	0.274	-4.07 (-9.07, 0.92)	0.111		
60-69 years	-4.54 (-7.77, -1.31)	0.006	-6.52 (-9.72, -3.31)	0.001	-9.04 (-13.35, -4.74)	0.001		
>=70 years	-8.51 (-12.73, -4.28)	0.001	-7.70 (-11.89, -3.51)	0.001	-12.71 (-18.49, -6.99)	0.001		
Gender								
Male	Reference Group							
Female	-5.64 (-7.84, -3.43)	0.001	-3.94 (-6.12, -1.75)	0.001	-3.64 (-6.57, -0.72)	0.015		
Marital Status								
Never married	Reference Group							
Currently married					6.48 (0.50, 12.47)	0.034		
Seprated/Divorced					-6.54 (-14.49, 1.04)	0.107		
Monthly Income								
>10000 PKR	Reference Group							
10000-20000 PKR	5.20 (-0.29, 10.71)	0.063					2.49 (-2.70, 7.69)	0.347
20000-30000 PKR	7.17 (1.71, 12.62)	0.011					3.61 (-1.54, 8.77)	0.170
30000-40000 PKR	8.32 (2.93, 13.71)	0.003					8.40 (3.32, 13.49)	0.001
>40000 PKR	6.46 (0.58, 12.33)	0.031					9.12 (3.67, 14.68)	0.001
Employment Status								
Employed	8.30 (6.02, 10.59)	0.001	9.09 (6.81, 11.37)	0.001	7.36 (4.34, 10.38)	0.001	4.76 (2.63, 6.89)	0.001
Unemployed	Reference Group							
Educational Status								
Illiterate	Reference Group							
Under secondary school	0.64 (-0.81, 2.67)	0.115	0.53 (-0.11, 2.29)	0.167				
Under Intermediate	1.65 (0.71, 5.43)	0.004	2.35 (0.87, 7.43)	0.001				
at least bachelors	3.24 (1.21, 7.58)	0.001	6.42 (2.93, 10.62)	0.001				

## Discussion

The available literature on multimorbidity was mainly from developed countries using databases from primary health care facilities [14]. However, limited studies are available on this topic in low and middle-income countries, where 80% of the burden of non-communicable diseases falls [14]. A small number of published articles on multimorbidity in middle and low-income countries are limited to a small number of public health care facilities that do not give an idea about the true situation of multimorbidity [9]. Besides this, a clear picture from private health care facilities lacks as most studies did not include private health care facilities and countries like Pakistan, where most people consult private primary health care centers for consultation. The current was conducted with the aim to identify the predictors of quality of life among patients with multimorbidity.

The quality of life of patients suffer from any condition is important as it provides significant ideas about the outcomes of treatment. According to World Health Organization, health is defined as "A state of complete physical, mental, and social wellbeing not merely the absence of disease or infirmity" [15]. Health-related quality of life studies are appropriate to understand the impact of various interventions on the patient's emotional, social, and physical wellbeing. The current study used WHOQOL-BREF for the assessment of the quality of life among patients with multimorbidity. The findings of this study have shown that factors associated significantly with quality of life including age, gender, monthly income, employment status, and educational level.

In our study, the highest score was reported in the physiological domain, while the lowest was reported in the environment domain. The findings of the current study are in contrast to the study conducted by Van Damme-Ostapowicz et al. using the same instrument to assess the quality of life in malaria patients [16]. This study found that the highest satisfaction score was reported in the social domain while the lowest was in the physical domain [16]. Our study has shown that younger patients have a better quality of life in contrast to the patients in the older age group. Similar findings have been reported in past studies [13]. This finding could be attributable to the reason that older people may have a lesser tolerance for the sickness than younger people. Another factor could be that physical functioning has deteriorated as a result of increased age. Gender is also a significant factor that impacts the quality of life of patients with multimorbidity. Females have low satisfaction scores in three domains. The findings of this study are consistent with the results reported by Pati et al. [9]. In middle and low-income countries like Pakistan, females are more vulnerable to the impacts of gender inequality, due to which they are more likely to have poor quality of life than their counterparts. 

The quality of life of well-educated individuals in our study was better as compared to illiterate people because people with a higher level of education are more concerned about their wellbeing, and they have better knowledge about the management of the disease. Past studies have reported similar findings [17]. Therefore, awareness of patients can be an important strategy to prevent disease severity and enhance their quality of life. The current study has reported that the marital status of women is significantly associated with the social relationship domain of quality of life. It means that married people have a better quality of life as compared to unmarried people. Similar findings were also reported by Ha et al. [13].

Findings that multimorbidity is associated with poor quality of life have important implications for individuals with multimorbidity in low and middle-income countries. Population in middle and low-income countries are more likely to have poor quality of life due to lack of access to quality health care, lack of financial resources, and poor facilities. It is important for health care professionals at all levels, including primary, secondary, and tertiary health care levels, to work closely with individuals to enhance the capabilities of patients in order to enhance their independence and autonomy to control factors affecting the quality of their lives through proper assessment of all the factors that can affect the quality of life. In addition, enhancing the quality of life need to be an important objective of the treatment and management plan of patients with multimorbidity to make them more self-dependent so they can manage their disease well. It will lead to positive health outcomes for patients and for their families as well. 

Our study has certain limitations and strengths that need to be considered while interpreting the current study findings. First, it was a cross-sectional study, and therefore, it is limited to assess the association instead of the causality between the quality of life and other factors. Another limitation of the current study is that all were self-reported details and no data were taken from the clinical profiles of participants. One of the strengths of this study is it used WHOQOL-BREF to assess the quality of life. This instrument has been proved to be valid and reliable across 23 nations [18]. Secondly, this is one of the few studies in Pakistan that assess the quality of life of patients with multimorbidity. Thirdly, this study included the enrollment of samples from different public health care facilities. Furthermore, the population's demographics are very representative of other communities in poor countries, making them useful outside the immediate community. This argument is bolstered by the fact that our findings are comparable to those of previous studies conducted in underdeveloped nations.

## Conclusions

This study has shown the low quality of life among patients with multimorbidity living in Karachi, Pakistan. Employment status is the important factor affecting all the domains in quality of life. Older age was associated with lower quality of life in physical health, psychological health, and social relationships. Women with multimorbidity had lower satisfaction ratings in physical health, psychological health, and social relationships than males. The findings of this study had important implications for identifying distinct multimorbidity individuals who were at risk of a lower quality of life, and they emphasized the need for disease detection and treatment at an early stage. The study can also give important evidence for decision-makers when it comes to allocating health resources more efficiently, and health administrative departments can improve chronic disease management and monitoring while also boosting awareness about chronic disease prevention. In a prospective cohort study, future research should look into the relationship between more detailed multimorbidity patterns and quality of life.

## Appendices

                                                                                     ** Survey** **Questionnaire**

1) Participant gave consent

1- Yes

2- No

2) Any Chronic condition (Mark all that apply)

0- None

1- Phthisis

2- Depression

3- Anxiety

4- Dementia

5- Multiple sclerosis

6- Cancer,

7- Chronic kidney disease

8- Chronic obstructive pulmonary disease

9- Gallbladder and spleen disease

10- Stroke

11- Peripheral vascular disease

12- Coronary disease

13- Gout

14- Gastroenteritis

15- Dyslipidemia

16- Diabetes mellitus

17- Bones diseases

18- Chronic pain

19- Hypertension

20- Other

Please Specify.....................

- If a participant has at least two diseases from the above list, then enroll in the study

3) Age

……… in years

4)  Gender

1- Male

2- Female

5) Marital Status

1- Single

2- Married

3- Widowed/Separated

6) Ethnicity

1-  Sindhi

2- Punjabi

3- Baluchi

4- Pashtu

5- Urdu

6- Other

7) Education

……….. In Years

0 if Never got any formal education

8) Current Employment status

1- Employed

2- Unemployed

9) Monthly Family income

…………….. in PKR

Question to assess quality of life

The following questions ask about how much you have experienced certain things in the last four weeks.

1a- To what extent do you feel that physical pain prevents you from doing what you need to do?

1- Not at all

2- A little

3- A moderate amount

4- Very Much

5- Extremely

2a- How much do you need any medical treatment to function in your daily life?

1- Not at all

2- A little

3- A moderate amount

4- Very Much

5- Extremely

3a- How much do you enjoy life?

1- Not at all

2- A little

3- A moderate amount

4- Very Much

5- Extremely

4a- To what extent do you feel your life to be meaningful?

1- Not at all

2- A little

3- A moderate amount

4- Very Much

5- Extremely

5a- How well are you able to concentrate?

1- Not at all

2- A little

3- A moderate amount

4- Very Much

5- Extremely

6a- How safe do you feel in your daily life?

1- Not at all

2- A little

3- A moderate amount

4- Very Much

5- Extremely

7a- How healthy is your physical environment?

1- Not at all

2- A little

3- A moderate amount

4- Very Much

5- Extremely

The following questions ask about how completely you experience or were able to do certain things in the last four weeks.

8a- Do you have enough energy for everyday life?

1- Not at all

2- A little

3- Moderately

4- Mostly

5- Completely

9a- Are you able to accept your bodily appearance?

1- Not at all

2- A little

3- Moderately

4- Mostly

5- Completely

10a- Have you enough money to meet your needs?

1- Not at all

2- A little

3- Moderately

4- Mostly

5- Completely

11a- How available to you is the information that you need in your day-to-day life?

1- Not at all

2- A little

3- Moderately

4- Mostly

5- Completely

12a- To what extent do you have the opportunity for leisure activities?

1- Not at all

2- A little

3- Moderately

4- Mostly

5- Completely

13a- How well are you able to get around?

 1- Very poor

2- poor

3- Neither good nor poor

4- good

5- Very good

14a- How satisfied are you with your sleep?

 1- Very dissatisfied

2- Dissatisfied

3- Neither satisfied or dissatisfied

4- Satisfied

5- Very satisfied

15a- How satisfied are you with your ability to perform your daily living activities?

 1- Very dissatisfied

2- Dissatisfied

3- Neither satisfied or dissatisfied

4- Satisfied

5- Very satisfied

16a- How satisfied are you with your capacity for work?

 1- Very dissatisfied

2- Dissatisfied

3- Neither satisfied or dissatisfied

4- Satisfied

5- Very satisfied

17a- How satisfied are you with yourself?

 1- Very dissatisfied

2- Dissatisfied

3- Neither satisfied or dissatisfied

4- Satisfied

5- Very satisfied

18a- How satisfied are you with your personal relationships?

 1- Very dissatisfied

2- Dissatisfied

3- Neither satisfied or dissatisfied

4- Satisfied

5- Very satisfied​​​​​​​

19a- How satisfied are you with your sex life?

 1- Very dissatisfied

2- Dissatisfied

3- Neither satisfied or dissatisfied

4- Satisfied

5- Very satisfied​​​​​​​

20a- How satisfied are you with the support you get from your friends?

 1- Very dissatisfied

2- Dissatisfied

3- Neither satisfied or dissatisfied

4- Satisfied

5- Very satisfied​​​​​​​

21a- How satisfied are you with the conditions of your living place?

 1- Very dissatisfied

2- Dissatisfied

3- Neither satisfied or dissatisfied

4- Satisfied

5- Very satisfied​​​​​​​

22a- How satisfied are you with your access to health services?

 1- Very dissatisfied

2- Dissatisfied

3- Neither satisfied or dissatisfied

4- Satisfied

5- Very satisfied​​​​​​​

23a- How satisfied are you with your transport?

 1- Very dissatisfied

2- Dissatisfied

3- Neither satisfied or dissatisfied

4- Satisfied

5- Very satisfied​​​​​​​

24a- How often do you have negative feelings such as blue mood, despair, anxiety, depression?

1- Never

2- Seldom

3- Quite often

4- Very often

5- Always

## References

[1] Valderas JM, Starfield B, Sibbald B, Salisbury C, Roland M (2009). Defining comorbidity: implications for understanding health and health services. Ann Fam Med.

[2] Walker V, Perret-Guillaume C, Kesse-Guyot E (2016). Effect of multimorbidity on health-related quality of life in adults aged 55 years or older: results from the SU.VI.MAX 2 cohort. PLoS One.

[3] Fortin M, Soubhi H, Hudon C, Bayliss EA, van den Akker M (2007). Multimorbidity's many challenges. BMJ.

[4] Brett T, Arnold-Reed DE, Popescu A (2013). Multimorbidity in patients attending 2 Australian primary care practices. Ann Fam Med.

[5] Marengoni A, Winblad B, Karp A, Fratiglioni L (2008). Prevalence of chronic diseases and multimorbidity among the elderly population in Sweden. Am J Public Health.

[6] Naz L, Ghimire U, Zainab A (2021). Behavioral factors associated with utilization of healthcare services among elderly in Pakistan: evidence from a nationally representative survey. BMC Geriatr.

[7] Fortin M, Bravo G, Hudon C, Lapointe L, Almirall J, Dubois MF, Vanasse A (2006). Relationship between multimorbidity and health-related quality of life of patients in primary care. Qual Life Res.

[8] Bao XY, Xie YX, Zhang XX, Peng X, Huang JX, Du QF, Wang PX (2019). The association between multimorbidity and health-related quality of life: a cross-sectional survey among community middle-aged and elderly residents in southern China. Health Qual Life Outcomes.

[9] Pati S, Swain S, Knottnerus JA, Metsemakers JF, van den Akker M (2020). Magnitude and determinants of multimorbidity and health care utilization among patients attending public versus private primary care: a cross-sectional study from Odisha, India. Int J Equity Health.

[10] Møller A, Bissenbakker KH, Arreskov AB, Brodersen J (2020). Specific measures of quality of life in patients with multimorbidity in primary healthcare: a systematic review on patient-reported outcome measures' adequacy of measurement. Patient Relat Outcome Meas.

[11] Smith AW, Reeve BB, Bellizzi KM (2008). Cancer, comorbidities, and health-related quality of life of older adults. Health Care Financ Rev.

[12] The WHOQOL Group (1998). Development of the World Health Organization WHOQOL-BREF quality of life assessment. Psychol Med.

[13] Ha NT, Duy HT, Le NH, Khanal V, Moorin R (2014). Quality of life among people living with hypertension in a rural Vietnam community. BMC Public Health.

[14] Pati S, Swain S, Hussain MA (2015). Prevalence and outcomes of multimorbidity in South Asia: a systematic review. BMJ open.

[15] Svalastog AL, Donev D, Jahren Kristoffersen N, Gajović S (2017). Concepts and definitions of health and health-related values in the knowledge landscapes of the digital society. Croat Med J.

[16] Van Damme-Ostapowicz K, Krajewska-Kułak E, Rozwadowska E, Nahorski WL, Olszański R (2012). Quality of life and satisfaction with life of malaria patients in context of acceptance of the disease: quantitative studies. Malar J.

[17] WHOQOL-HIV Group (20031). Preliminary development of the World Health Organsiation's Quality of Life HIV instrument (WHOQOL-HIV): analysis of the pilot version. Social Science & Medicine.

[18] Skevington SM, Lotfy M, O'Connell KA (2004). The World Health Organization's WHOQOL-BREF quality of life assessment: psychometric properties and results of the international field trial. A report from the WHOQOL group. Qual Life Res.

